This article has been retracted.

# circRNA LDLRAD3 Enhances the Malignant Behaviors of NSCLC Cells via the miR-20a-5p-SLC7A5 Axis Activating the mTORC1 Signaling Pathway

**DOI:** 10.1155/2022/2373580

**Published:** 2022-01-06

**Authors:** Yu Li, Guangle Qin, Jinyun Du, Peng Yue, Yanling Zhang, Na Hou

**Affiliations:** ^1^Department of ICU Medicine, Shandong Province Zibo No. 1 Hospital, Zibo 255200, Shandong, China; ^2^Emergency Department, Shandong Province Zibo No. 1 Hospital, Zibo 255200, Shandong, China; ^3^Department of Intensive Care, Boxing County Hospital of Traditional Chinese Medicine, Binzhou 256500, Shandong, China; ^4^Oncology Dept. II, Shandong Province Zibo No. 1 Hospital, Zibo 255200, Shandong, China

## Abstract

Circular RNA LDLRAD3 behaved as an oncogene in several malignancies, but its effects in NSCLC and the involvement of downstream molecules and activation of signaling pathways had not been fully reported. We planned to explore how LDLRAD3 facilitated the malignancy of NSCLC. QRT-PCR was performed to evaluate the expression levels of LDLRAD3, miR-20a-5p, and SLC7A5 in NSCLC tissues and cells. si-LDLRAD3 was transfected to A549 and H1299 cells to knock down intrinsic LDLRAD3 to determine its oncogenic roles. CCK-8 assay and transwell assay were executed to assess cell proliferative, migrative, and invasive abilities. Dual-luciferase reporter (DLR) assay was manipulated to verify the ENCORI-predicted relationships between LDLRAD3 and miR-20a-5p and between miR-20a-5p and SLC7A5. Western blot, immunofluorescent assay, and immunohistochemistry were applied to explore the expression levels of SLC7A5, and the levels of mTORC1 pathway-related proteins were evaluated using western blot. Rescue experiments were conducted by transfecting si-LDLRAD3, miR-20a-5p inhibitor, and si-SLC7A5 to explore the influence of the LDLRAD3-miR-20a-5p-SLC7A5 axis on the malignant behaviors of NSCLC cells. The expression levels of LDLRAD3 and SLC7A5 were boosted, whereas miR-20a-5p was impeded in NSCLC tissues and cell lines. Knockdown of LDLRAD3 weakened the proliferation, migration, and invasion of A549 and H1299 cells. LDLRAD3 was verified to sponge miR-20a-5p and miR-20a-5p targeted SLC7A5. LDLRAD3 activated the mTORC1 singling pathway via the miR-20a-5p-SLC7A5 axis to strengthen the malignant properties of A549 and H1299 cells. We concluded that LDLRAD3 exerted oncogenic effects via the miR-20a-5p-SLC7A5 axis to activate the mTORC1 signaling pathway in NSCLC. Our findings enlightened that LDLRAD3 could become a potential therapeutic target in the treatment and management of NSCLC.

## 1. Introduction

Lung cancer is the most dangerous killer and the global leading factor of cancer-related deaths [1]. In China, it ranks the highest morbidity and mortality in the past ten years [2]. In addition, lung cancer can be classified into small-cell lung cancer (SCLC) and non-small-cell lung cancer (NSCLC) based on histopathology and NSCLC accounts for 85% of cases [3]. Currently, the lack of precise molecular targets for the treatment and monitoring methods against metastasis, and recurrence has become a serious challenge in NSCLC therapy [4]. Therefore, it is high time to find more reliable molecules to alleviate the burden of cancer monitoring.

Circular RNA (circRNA) with a closed, continuous loop structure is a class of widely expressed noncoding RNA [5]. It has high sensitivity and tissue-specificity and can act as a molecular regulator to exert different mediatory functions in different cancers [6]. For instance, it can act as microRNA sponges, interact with RNA binding proteins, regulate gene expressions, and control translation [7]. Tian et al. have reviewed the clinical values and the potential of circRNAs as biomarkers in the treatment of gastric cancer [8]. In NSCLC, several aberrantly expressed circRNAs have been reported, such as low expressed ITCH, ZEB1.5 and highly expressed CMPKI, PRKCI, and HIPK3 [7]. circRNA low-density lipoprotein receptor class A domain containing 3 (LDLRAD3) is highly expressed in NSCLC tissues, and it can sponge miR-137 to promote SLC1A5 expression, thus boosting the proliferation of A549 and H1299 cells and impeding cell apoptosis [9]. Besides this, LDLRAD3 also accelerates pancreatic cancer progression via the miR-137-PTN axis [10] and promotes metastasis of gastric cancer through the miR-224-5p-NRP2 axis [11]. Therefore, we hypothesize that LDLRAD3 should be an oncogenic molecule and plan to look for the potential target of LDLRAD3 in NSCLC cells due to its regulatory roles in cancer by sponging microRNAs (miRNAs) in a competing endogenous RNA-dependent manner [12].

miRNA is also a type of noncoding RNA that degrades their target mRNAs or suppresses translation complementarily [13]. During cancer progression, miRNAs behave like oncogenes or tumor suppressors, and they are abnormally expressed in different cancers [13]. For instance, miR-20a-5p is low expressed in NSCLC tissues and exerts antitumor roles via inhibiting the RRM2-mediated PI3K/Akt signaling pathway [14]. It also retards postoperative metastasis of liver cancer via blocking HGF/ERBB3-NF*κ*B pathway [15]. As miRNAs can act as mRNA sponges in the mediation of NSCLC progression [16], we plan to explore more complementary target mRNA of miR-20a-5p in NSCLC cells.

SLC7A5 is a sodium-independent transporter and acts as an amino acid exchanger by transporting large neutral amino acids such as leucine, phenylalanine, and tryptophan by exchange with intracellular glutamine. SLC7A5 is located in 16q24.2, and its functions in supplying amino acids to cancer cells and maintaining intracellular leucine [17]. It also supplies amino acids to cancer cells and stimulates the mTORC1 signaling pathway, which is an essential pathway related to cancer cell proliferation and invasive behaviors [18]. SLC7A5 is widely expressed in many human cancers and various cancer cell lines; researches have demonstrated that SLC7A5 is highly expressed in different tumors, such as breast cancer [18], oral cancer [19], and NSCLC tissues [20]. In addition to this, SLC7A5 is coexpressed with the glutamine transporter, SLC1A5, in many cancers suggesting a functional coupling of these transporters in supporting tumor progression [21]. In colon cancer and NSCLC, knockdown of SLC7A5 can block the mTORC1 pathway to deter cancer cell proliferation and tumor growth [22]. Another example is that SLC7A5 can be sponged by miR-126, and this process will inhibit cancer progression [23].

Here, we are motivated to connect LDLRAD3, miR-20a-5p, SLC7A5, and the mTORC1 signaling pathway in NSCLC cells and use qRT-PCR, western blot, immunofluorescent assay, DLR assay, and transwell assays to investigate their relationships and the involvement of potential mechanisms in the mediation of the malignant behaviors of NSCLC cells to look for a novel potential therapeutic target for the treatment and management of NSCLC.

## 2. Material and Methods

### 2.1. Tissue Samples

This research was approved by the Shandong Province Zibo No. 1 Hospital, and the protocol followed the Declaration of Helsinki. A total of 30 NSCLC tissues and their corresponding tumor-adjacent normal tissues were resected and collected in our study. The informed written consent was signed and collected from all patients. None of them received any radiochemotherapy before resection. The cancerous tissues were examined microscopically and staged based on the 7^th^ edition of TNM staging from AJCC (USA). The survival data were continuously tracked for 60 months.

### 2.2. Cell Culture

4 human NSCLC cell lines (A549, H1299, HCC827, and Calu-3) and 1 human bronchial epithelial cell line (BEAS-2B) were ordered from Procell (China) and cultured appropriately. In detail, A549 was grown in Ham's F-12K (Procell, China). H1299 and HCC827 were cultivated in RPMI-1640 (Procell, China), whereas Calu-3 was inoculated in MEM (Gibco, USA). All the media mentioned above were supplemented with 10% FBS (Procell, China) and 1% p/s (Procell, China). BEAS-2B was maintained in BEGM (Procell, China). All of them were maintained in an incubator (MG80, Kuansons, China) containing 5% CO_2_ at 37°C.

### 2.3. Transfection

48 h before transfection, A549 and H1299 cells were transferred into 6-well plates. To knock down endogenous LDLRAD3, miR-20a-5p, and SLC7A5, the cells at 70–80% confluence were transfected by small interfering RNAs (siRNAs) (si-NC and si-LDLRAD3; inhibitor-NC and miR-20a-5p inhibitor; si-NC and si-SLC7A5). The oligos sequences were supplied by OriGene (China). The transfection process was conducted with in vitro RNA kit (InvivoGen, China) according to the protocol.

### 2.4. qRT-PCR

The MolPure Cell RNA Kit (Yeasen, China) was chosen for the extraction and purification of RNA from NSCLC tissues and cells. RNAs shorter than 200 nucleotides were extracted with MolPure Cell/Tissue miRNA Kit (Yeasen, China). The reverse transcription was executed using the Hifair III 1st-Strand cDNA Synthesis Kit with gDNA digester plus (Yeasen, China). To evaluate the expression levels of LDLRAD3, miR-20a-5p, and SLC7A5, the qRT-PCR process was achieved with the Q960 PCR instrument (Dinai, China) using the PC46-THERMOscript SYBR Green qRT-PCR Kit (Aidlab, China). The primer sequences were as follows: LDLRAD3 forward: 5′-CTT GCT GGA CCA GAG AAC ACA TG-3′, reverse: 5′-CAT GAG GTT GTT CCG CTT CCC A-3′; miR-20a-5p forward: 5′-UAC AGC GCA GAC AGU GCA GCU AG-3′, reverse: 5′-CUA GCU GAA CUA CGC ACU GUA-3′; SLC7A5 forward: 5′-GAA GTC ACC AAG TAC ACT GGA TGT-3′, reverse: 5′-GAA GTA GTC CAG GTT GGT CAG A-3′; U6 forward: 5′-GGA AGC TTG TCA TCA ATG GAT ATC-3′, reverse: 5′-TGA TGA CCC TTT TGG CTC CAA C-3′; and *β*-actin forward: 5′-CAT TGT TAC CAA CTG GGA CGA CAT-3′, reverse: 5′-GCC TCG GTG AGC AGC TTA CA-3′. The relative expression levels of LDLRAD3 and SLC7A5 mRNA were normalized with *β*-actin, and the relative expression level of miR-20a-5p was normalized with U6 via the 2^−ΔΔCt^ method.

### 2.5. Western Blot

Proteins were extracted with Nuclear and Cytoplasmic Protein Extraction Kit (Yeasen, China), and their concentrations were checked with BCA Protein Quantification Kit (Yeasen, China). After being separated using SDS-PAGE with PAGE Gel Quick Preparation Kit (12.5% and 10%) (Yeasen, China) and transferred onto the PVDF membrane (GE, USA), the unreacted sites were blocked with 5% skim milk (Beyotime, China) for 2 h and the primary antibodies against SLC7A5 (1 : 200, goat, ab99419), *β*-actin (1 : 500, goat, ab8229; 1 : 1000, rabbit, ab8227), p-mTOR (phospho-S2448, 1 : 1000, rabbit, ab109268), mTOR (1 : 1000, rabbit, ab32028), p-S6K1 (phospho-S424, 1 : 500, rabbit, ab131436), S6K1 (1 : 5000, rabbit, ab32529), p-4EBP (1 : 500, rabbit, ab47365), and 4EBP (1 : 2000, rabbit, ab32024) (Abcam, USA) were added and the samples were incubated at 4°C for 12 h. After being rinsed three times with TBST (Yeasen, China), the secondary HRP-conjugated donkey anti-goat antibody (1 : 1000, ab6885) or goat anti-rabbit antibody (1 : 2000, ab6721) (Abcam, USA) was administrated to the membrane and maintained for 1 h at room temperature. Next, the bands were washed with TBS-T and visualized using the 4CN HRP kit (Leagene, China). The relative expression levels were obtained via ImageJ 1.53f (NIH, USA).

### 2.6. Immunohistochemistry Assay

The tissue specimens were fixed, embedded, and sliced. After deparaffinization and rehydration, the primary rabbit antibodies against SLC7A5 (1 : 500, ab208776), p-mTOR (phospho-S2448, 1 : 100, ab109268), p-S6K1 (phospho-S424, 1 : 100, ab131436), and p-4EBP (1 : 100, ab47365) were added, and the specimens were incubated for 12 h at 4°C. Then, the secondary HRP-conjugated goat anti-rabbit antibody (1 : 1000, ab6721) (Abcam, USA) was added and incubated for 1 h at room temperature. Enhanced HRP-DAB Chromogenic Kit (Tiangen, China) was administrated to localize the antigens in the tissue samples.

### 2.7. Immunofluorescent Assay

The cells were fixed with 4% formaldehyde (Solarbio, China) for 0.5 h and then incubated with 0.1% Triton X-100 (Tiangen, China) for 15 min. Then, 5% BSA (Solarbio, China) was applied for blocking the unreacted sites for 0.5 h, and the primary rabbit antibody against SLC7A5 (1 : 500, ab208776) was administrated for 12 h at 4°C. Then, the secondary goat anti-rabbit antibody conjugated to Alexa Fluor 488 (1 : 200, ab150077, Abcam, USA) was administrated for 1 h at room temperature. The images were captured by the CKX53 microscope (Olympus, Japan) with an emission wavelength of 495 nm and an emission wavelength of 519 nm [24].

### 2.8. DLR Assay

The interactions between LDLRAD3 and miR-20a-5p or miR-20a-5p and SLC7A5 were indicated by ENCORI. The oligo sequence of LDLRAD3 and 3′-UTR of SLC7A5 carrying the wild type or mutant binding sites of miR-20a-5p and were amplified using Q960 PCR instrument (Dinai, China) and inserted into pmirGLO Dual-Luciferase miRNA Target Expression Vector (Promega, USA) to create the plasmids (LDLRAD3-WT and LDLRAD3-MT; SLC7A5-WT and SLC7A5-MT). The mimic-NC and miR-20a-5p mimic were cotransfected with the above vectors using Hieff Trans Liposomal Transfection Reagent kit (Yeasen, China), and the luciferase activity was measured with DLR Gene Assay Kit (Yeasen, China) and GloMax 20/20 Luminometer (Promega, USA). The luminescence activity of firefly luciferase substrate was normalized to Renilla luciferase substrate [25].

### 2.9. CCK-8 Assay

A549 and H1299 cells were seeded into 96-well plates at 1 × 10^4^ cells/well and maintained for different periods. After that, 10 *μ*l of CCK-8 solution was administrated into each well and incubated for 2 h and cell proliferation was determined using Cell Counting Kit (AbMole, China). The absorbances were measured by the DR-3518G microplate reader (Diatek, China) at 450 nm [26].

### 2.10. Transwell Migration and Invasion Assay

Transfected A549 and H1299 cells were inoculated in the 500 *μ*l medium in the upper chamber of 24-well transwell plates (Corning, USA) containing 8 *µ*m pore at a density of 1 × 10^5^ cells/well. For the invasion assay, the upper chamber was precoated with 150 *μ*L/cm^2^ Matrigel Basement Membrane Matrix (Solarbio, China). Besides, 1 mL medium with 15% FBS (Solarbio, China) was supplied in the lower chamber and the cells were incubated for 48 h. The upper chamber was supplied with serum-free RPMI-1640 (Procell, China). The cells that remained at the upper surface of the membrane were removed, and the migrated or invaded cells below the membrane were fixed with 4% paraformaldehyde (Solarbio, China) for 0.5 h and stained using 10% crystal violet (Solarbio, China) for 0.5 h then observed using CKX53 microscope (Olympus, Japan).

### 2.11. Statistical Analysis

The experiments were performed in triplicate. Data were expressed as mean ± SD. Prism 8.3.0 (GraphPad, USA) which was a popular software for statistical analysis and graph plotting was selected for data processing and graph plotting. The differences between the two groups were assessed through the Student *t*-test and/or among the multiple groups were assessed using one-way analysis of variance (ANOVA). The correlation between LDLRAD3 and miR-20a-5p and that between miR-20a-5p and SLC7A5 were analyzed with Spearman's rank-order correlation test. The survival rates of patients were determined using the Kaplan–Meier survival curve. *P* < 0.05 was recognized as statistically significant.

## 3. Results

### 3.1. High LDLRAD3 Expression in NSCLC Tissues and Cells and Exerted Oncogenic Roles

To evaluate the expression level of LDLRAD3 in 30 NSCLC tissues (I + II, *n* = 16; III + IV, *n* = 14) and paired normal tissues (*n* = 30), qRT-PCR was performed, and it was shown that its expression level was higher in cancerous tissues compared with the corresponding tumor-adjacent normal tissues (*P* < 0.01) and the higher level of LDLRAD3 was detected in the cancerous tissues of III + IV grades compared with I + II grades (*P* < 0.01) (Figure 1(a)). Besides, the patients of the high LDLRAD3 level group (higher than the median, *n* = 13) had a lower survival rate than the low LDLRAD3 level group (*n* = 17) (*P* < 0.05) (Figure 1(b)). Thereafter, we measured the expression level of LDLRAD3 in 4 human NSCLC cell lines and a bronchial epithelial cell line using qRT-PCR. The results reported that all the NSCLC cell lines expressed higher levels of LDLRAD3 than BEAS-2B. In addition to this, A549 and H1299 expressed relatively higher levels of LDLRAD3 among these 4 NSCLC cell lines (Figure 1(c)). Therefore, to determine the roles of LDLRAD3, they were selected to establish the LDLRAD3 knockdown cell models via transfection of siRNAs to knock down the endogenous LDLRAD3. The high transfection efficiency was verified with qRT-PCR (Figure 1(d)). After that, the results of the CCK-8 assay (*P* < 0.01) (Figure 1(e)) indicated that the proliferative abilities of A549 and H1299 cells were inhibited after the knockdown of LDLRAD3, which was reflected by the changes of absorbance. Then, using transwell assays, it was detected that knockdown of LDLRAD3 lessened the migrative (*P* < 0.01) (Figure 1(f)) and invasive (*P* < 0.01) (Figure 1(g)) abilities of both cell lines. And A549 exerted stronger migrative and invasive abilities than H1299. These results exhibited that knockdown of LDLRAD3 diminished the malignant behaviors of NSCLC cells.

### 3.2. LDLRAD3 Sponged miR-20a-5p

We evaluated the expression level of miR-20a-5p in 30 pairs of NSCLC tissues (I + II, *n* = 16; III + IV, *n* = 14) and paired normal tissues with qRT-PCR and found that the cancerous tissues expressed a lower level of miR-20a-5p than tumor-adjacent normal tissues (*P* < 0.05), and the cancerous tissues of I + II grades owned a lower expression level of miR-20a-5p compared with the tissues of III + IV grades (*P* < 0.01) (Figure 1(h)). Then, we conducted Spearman's correlation test and obtained that the expression level of miR-20a-5p was negatively correlated with the expression level of LDLRAD3 in cancerous tissues (Figure 1(i)). Next, the data from ENCORI predicted that LDLRAD3 could bind to miR-20a-5p (Figure 1(j)). This prediction was confirmed by the DLR assay, which showed that the application of miR-20a-5p mimics weakened the luciferase activity of LDLRAD3-WT group, but not the LDLRAD3-MT group (*P* < 0.01), which confirmed that LDLRAD3 could bind to miR-20a-5p (Figure 1(k)). Thereafter, we explored the expression level of miR-20a-5p in the transfected A549 and H1299 cell lines and found that the expression level of miR-20a-5p was higher in the si-LDLRAD3 group compared with the blank group and si-NC group (all *P* < 0.01) (Figure 1(l)). These results above pointed out that LDLRAD3 could sponge miR-20a-5p and knockdown of LDLRAD3 boosted the expression level of miR-20a-5p.

### 3.3. LDLRAD3 Targeted miR-20a-5p to Promote SLC7A5 Expression

QRT-PCR was performed to evaluate the mRNA expression level of SLC7A5 in the paired cancerous and normal tissues, and it was indicated that its expression level was higher in cancerous specimens than normal tissues (*P* < 0.05) and a higher expression level of SCL7A5 was detected in the cancerous tissues of III + IV grades than I + II grades (*P* < 0.01) (Figure 2(a)). Besides, the results of western blot (*P* < 0.01) (Figure 2(b)) and immunohistochemistry (Figure 2(c)) also presented similar findings. Thereafter, we executed Spearman's correlation test and explored that in the cancerous tissues, the expression level of miR-20a-5p was negatively correlated with SLC7A5 (*P* < 0.01) (Figure 2(d)), and we also obtained a positive correlation between the expression levels of LDLRAD3 and SLC7A5 in cancerous tissues (*P* < 0.01) (Figure 2(e)). Using ENRORI database, we found a predicted binding site between miR-20a-5p and 3′-UTR OF SLC7A5 (Figure 2(f)), and subsequently, this binding relationship was verified by DLR assay. The results proved that miR-20a-5p mimics dropped the relative luciferase activity of the SLC7A5-WT group, but not the SLC7A5-MT group (*P* < 0.01), which indicated that miR-20a-5p could bind to SCL7A5 mRNA (Figure 2(g)). Next, the miR-20a-5p inhibitor was transfected to A549 and H1299 cells, and the transfection efficiency was verified with qRT-PCR (Figure 2(h)). Afterward, to determine the mediatory roles of LDLRAD3 and miR-20a-5p in the expression level of SLC7A5, these two cell lines (A549 and H1299) were cotransfected with si-LDLRAD3 and miR-20a-5p inhibitor. The results of qRT-PCR exhibited that knockdown of LDLRAD3 by siRNA reduced the expression level of SLC7A5, whereas the transfection of miR-20a-5p inhibitor could partially counteract the effect of si-LDLRAD3 on the expression level of SLC7A5 (*P* < 0.01) (Figure 2(i)). Then, the results of western blot and immunofluorescent assay were consistent with the results of qRT-PCR (*P* < 0.01) (Figures 2(j)–2(k)). These findings above manifested that LDLRAD3 targeted miR-20a-5p to enhance the expression level of SLC7A5.

### 3.4. LDLRAD3 Activated mTORC1 Pathway to Facilitate Proliferation, Migration, and Invasion of NSCLC Cells via miR-20a-5p-SLC7A5 Axis

To explore the activation of the mTORC1 signaling pathway in the NSCLC tissues and normal tissues, immunohistochemistry was operated, and the representative results showed that the cancerous tissues expressed higher levels of p-mTOR, p-S6K1, and p-4EBP in comparison to normal tissues which indicated that the mTORC1 pathway was activated in NSCLC (Figure 3(a)). Then, A549 and H1299 cells were divided into 7 groups (Blank, si-NC + inhibitor-NC, si-LDLRAD3 + inhibitor-NC, si-NC + miR-20a-5p inhibitor, si-LDLRAD3 + miR-20a-5p inhibitor, si-LDLRAD3 + miR-20a-5p inhibitor + si-NC, and si-LDLRAD3 + miR-20a-5p inhibitor + si-SLC7A5) and cotransfected respectively to determine the roles of LDLRAD3-miR-20a-5p-SLC7A5 axis on the activation of the mTORC1 pathway. The results of western blot reported that knockdown of LDLRAD3 suppressed this pathway via reduction of the phosphorylation levels of mTOR, S6K1, and 4EBP, while knockdown of miR-20-5p stimulated this pathway. Moreover, the effects of transfecting miR-20-5p inhibitor could be completely reversed by transfection of si-SLC7A5 in both A549 and H1299 cell lines (*P* < 0.05 and *P* < 0.01) (Figure 3(b)).

Next, to investigate whether LDLRAD3 had oncogenic influences via the miR-20a-5p-SLC7A5 axis and the activation of the mTORC1 pathway, the proliferative, migrative, and invasive abilities of cotransfected A549 and H1299 cell lines were tested using CCK-8 assay and transwell assay. It was testified by the CCK-8 assay that knockdown of LDLRAD3 hampered the proliferative abilities of both cell lines; the impact of si-LDLRAD3 could be partially neutralized by miR-20a-5p inhibitor. And the promotive roles of miR-20a-5p inhibitor on cell proliferation were reversed by transfection of si-SLC7A5 (*P* < 0.01) (Figure 3(c)). Besides, similar results were obtained from the transwell assay. In detail, transfection of si-LDLRAD3 lessened the migrative and invasive abilities of NSCLC cells while these abilities were uplifted by miR-20a-5p inhibitor. And the effect of transfecting miR-20a-5p inhibitor was completely counteracted by transfection of si-SLC7A5 (*P* < 0.05 and *P* < 0.01) (Figures 3(d) and 3(e)). These consequences above indicated that LDLRAD3 ignited the mTORC1 signaling pathway through the miR-20a-5p-SLC7A5 axis to enhance the malignant behaviors of NSCLC cells.

## 4. Discussion

Lung cancer has become the most common incident cancer and the most dangerous killer in China, and the high metastatic and recurrent rates had become major problems of national public health [2]. Currently, the lack of reliable molecules for the monitoring and therapy of NSCLC which accounted for the majority of lung cancer cases inspired the researchers to focus on the discovery of novel therapeutic targets [27]. A recent article had reviewed that circRNAs showed tumor-regulatory roles in NSCLC progression via different mechanisms and they were expected to become potential diagnostic biomarkers for NSCLC [23]. For instance, the expression level of circular RNA FOXO3 was downregulated in NSCLC tissues, and it acted as a tumor suppressor gene to inhibit cell proliferation and invasion via sponging miR-155 in NSCLC cells [16]. Another example was circular RNA HIPK3, which was highly expressed in NSCLC tissues; it behaved as an oncogene to enhance the proliferation of NSCLC cells through the miR-379-IGF1 axis [8]. Here, we reported that the expression level of LDLRAD3 was higher in NSCLC tissues and cultivated cell lines in comparison to normal tissues and a bronchial epithelial cell line, which was consistent with Xue et al.'s research [9]. Besides this, our findings also indicated that A549 and H1299 cell lines had higher expression levels of LDLRAD3 than HCC827 and Calu-3. In addition, we also found a discrepancy between Xue et al.'s article [9] and our outcomes. In their results, A549 owned a higher level of LDLRAD3 than H1299, but we got a contrary result using qRT-PCR. Furthermore, knockdown of LDLRAD3 showed suppressive roles on the proliferation, migration, and invasion of A549 and H1299 cells. And this part of the results was consistent with Xue et al.'s study [9], which also used A549 and H1299 cell lines.

In NSCLC tissues and cells, the expression level of miR-20a-5p was downregulated, and it has been reported that it has tumor-suppressive roles, such as inhibition of tumor growth and angiogenesis *in vivo* and suppression of NSCLC cell proliferation, endothelial cells migration, and tube formation *in vitro* [14]. Our findings were consistent with this study. In our study, through qRT-PCR, it was indicated that the expression level of miR-20a-5p was diminished in NSCLC tissues and cultivated NSCLC cell lines in contrast to normal tissues and bronchial epithelial cell lines. Besides that, miR-20a-5p exhibited anticancer effects in different cancers. For instance, it inhibits EMT and the invasion of endometrial cancer cells via sponging STAT3 [12]. Another example is that in breast cancer cells, lncRNA HOTAIR could target miR-20a-5p to weaken its antitumor effects, such as inhibition of cell propagation and metastasis and facilitation of cell apoptosis [28]. In the present study, we identified that miR-20a-5p was targeted by LDLRAD3 and it was also complimentary with SLC7A5 to reduce its expression to show the tumor-regulatory roles of the LDLRAD3-miR-20a-5p-SLC7A5 axis, such as the control of cell proliferation, migration, and invasion of A549 and H1299 cells.

SLC7A5 is an L-type amino acid transporter 1, and the upregulated expression level of SLC7A5 was associated with high-grade tumors and metastasis of different cancer cells [29]. In our study, it was found that its expression level was higher in NSCLC tissues than normal tissues and knockdown of SLC7A5 impeded the malignant behaviors of NSCLC cells. Our finding was consistent with Imai et al.'s study [30], which also proposed that inhibition of SLC7A5 expression would show antitumor activity in NSCLC cells. Furthermore, SLC7A5 was a potential biomarker that presented tumorigenic influences through activation of its downstream mTORC1 signaling pathway. In detail, Elorza et al. have reported that HIF-1*α* could activate the mTORC1 pathway through upregulation of the expression level of SLC7A5 [31]. Our findings verified that knockdown of SLC7A5 could inhibit the phosphorylation of the mTORC1 pathway to retard the progression of NSCLC, which was consistent with Cormerais et al.'s results [32]. Moreover, the activated mTORC1 pathway had oncogenic roles in NSCLC [33], and our results also indicated that the regulation of the mTORC1 pathway by the LDLRAD3-miR-20a-5p-SLC7A5 axis was associated with malignant behaviors of NSCLC cells.

## 5. Conclusion

To conclude, we explored the oncogenic roles of circRNA LDLRAD3 in NSCLC in this research. It promotes the proliferative, migrative, and invasive abilities of A549 and H1299 cell lines via the miR-20a-5p-SLC7A5 axis to activate the mTORC1 signaling pathway. Besides that, the roles of LDLRAD3 as a therapeutic target for NSCLC needed to be continuously investigated in vivo and a special mTORC1 inhibitor was required to be selected to confirm the activation of this pathway by the LDLRAD3-miR-20a-5p-SLC7A5 axis. Our current results discovered a novel potential therapeutic target for the treatment and management of NSCLC and provided the theoretical basis for future studies.

## Figures and Tables

**Figure 1:** LDLRAD3 exerted oncogenic roles and it sponged miR-20a-5p. (a) The expression level of LDLRAD3 in NSCLC tissues and tumor-adjacent normal tissues was analyzed by qRT-PCR. (b) The survival time of patients with the LDLRAD3 expression level was higher or lower than the median. (c) The expression level of LDLRAD3 in NSCLC cell lines and a normal cell line was analyzed by qRT-PCR. (d) The expression level of LDLRAD3 in transfected A549 and H1299 cell lines was analyzed by qRT-PCR. (e) The proliferation of transfected cells was analyzed by CCK-8 assay. (f) The migration of cells was analyzed by transwell assay. (g) The invasion of cells was analyzed by transwell assay. (h) The expression level of miR-20a-5p in NSCLC tissues and tumor-adjacent normal tissues was analyzed by qRT-PCR. (i) The correlation between the expression levels of LDLRAD3 and miR-20a-5p in NSCLC tissues was analyzed by Spearman's correlation test. (j) The binding site of LDLRAD3 on miR-20a-5p was predicted by ENCORI. (k) The binding relationship between LDLRAD3 and miR-20a-5p was verified by the DLR assay. (l) The expression level of miR-20a-5p in transfected A549 and H1299 cell lines was analyzed by qRT-PCR. ^*∗*^*P* < 0.05 and ^*∗∗*^*P* < 0.01.

**Figure 2:** LDLRAD3 sponged miR-20a-5p to promote SLC7A5 expression. (a) The expression level of SLC7A5 mRNA was analyzed by qRT-PCR. (b) The expression level of SLC7A5 proteins was analyzed by western blot. (c) The expression level of SLC7A5 proteins was analyzed by immunohistochemistry. Scale bars: 50 *μ*m. (d) The correlation between the expression levels of miR-20a-5p and SLC7A5 in NSCLC tissues was analyzed by Spearman's correlation test. (e) The correlation between the expression levels of LDLRAD3 and SLC7A5 in NSCLC tissues was analyzed by Spearman's correlation test. (f) The binding site of miR-20a-5p on SLC7A5 was predicted by ENCORI. (g) The binding relationship between miR-20a-5p and SLC7A5 was verified by the DLR assay. (h) The expression level of miR-20a-5p in transfected A549 and H1299 cell lines was analyzed by qRT-PCR. (i) The expression level of SLC7A5 mRNA in cotransfected cells was analyzed by qRT-PCR. (j) The expression level of SLC7A5 protein in cotransfected cells was analyzed by western blot. (k) The expression level of SLC7A5 protein in cotransfected cells was analyzed by immunofluorescent assay. Scale bars: 50 *μ*m. ^*∗*^*P* < 0.01 and ^*∗∗*^*P* < 0.01.

**Figure 3:** LDLRAD3 activated the mTORC1 pathway to facilitate malignant behaviors of NSCLC cells via the miR-20a-5p-SLC7A5 axis. (a) The phosphorylation levels of proteins were analyzed by immunohistochemistry. Scale bars: 50 *μ*m. (b) The expression levels and phosphorylation levels of proteins in cotransfected cells were analyzed by western blot. (c) The proliferation of cotransfected cells was analyzed by CCK-8 assay. (d) The migration of cotransfected cells was analyzed by transwell assay. Scale bars: 100 *μ*m. (e) The invasion of cotransfected cells was analyzed by transwell assay. Scale bars: 5 *μ*m. ^*∗*^*P* < 0.05 and ^*∗∗*^*P* < 0.01.

## Data Availability

The simulation experiment data used to support the findings of this study are available from the corresponding author upon request.
